# Modification of Glycosylation Mediates the Invasive Properties of Murine Hepatocarcinoma Cell Lines to Lymph Nodes

**DOI:** 10.1371/journal.pone.0065218

**Published:** 2013-06-20

**Authors:** Zhaohai Zhang, Jie Sun, Lihong Hao, Chunqing Liu, Hongye Ma, Li Jia

**Affiliations:** 1 Department of Basic Laboratory Medicine, College of Laboratory Medicine, Dalian Medical University, Dalian, Liaoning Province, China; 2 Liaoning International Travel Health Care Center, Dalian, Liaoning Province, China; 3 Department of Histology and Embryology, Dalian Medical University, Dalian, Liaoning Province, China; INRS, Canada

## Abstract

Among the various posttranslational modification reactions, glycosylation is the most common, and nearly 50% of all known proteins are thought to be glycosylated. In fact, changes in glycosylation readily occur in carcinogenesis, invasion and metastasis. This report investigated the modification of glycosylation mediated the invasive properties of Hca-F and Hca-P murine hepatocarcinoma cell lines, which have high, low metastatic potential in the lymph nodes, respectively. Analysis revealed that the N-glycan composition profiling, expression of glycogenes and lectin binding profiling were different in Hca-F cells, as compared to those in Hca-P cells. Further analysis of the N-glycan regulation by tunicamycin (TM) application or PNGase F treatment in Hca-F cells showed partial inhibition of N-glycan glycosylation and decreased invasion both *in vitro* and *in vivo.* We targeted glycogene ST6GAL1, which was expressed differently in Hca-F and Hca-P cells, and regulated the expression of ST6GAL1. The altered levels of ST6GAL1 were also responsible for changed invasive properties of Hca-F and Hca-P cells both *in vitro* and *in vivo*. These findings indicate a role for glycosylation modification as a mediator of tumor lymphatic metastasis, with its altered expression causing an invasive ability differentially.

## Introduction

It is well known that glycosylation affects many physicochemical properties of glycoproteins. Thus, modified oligosaccharides affect protein folding and stability, and as a result, regulate many physiological and pathological events, including cell growth, migration, differentiation, and tumor metastasis [1]–[4]. Therefore, it is not surprising that aberrant glycosylation patterns can be considered to have great potential as therapeutic targets or clinical biomarkers for early detection, diagnosis and monitoring of cancer treatment.

Cancer metastasis shows a multi-step process. Specific changes in the glycosylation pattern of cell surface glycoproteins have been shown to correlate with the enhancement of the metastatic efficiency of tumor cells [5]. In particular, N-glycans cover the most outer surface and thus should be the first molecules to be contacted when cells interact with each other. There is ample evidence that altered N-glycosylation patterns are present on tumor cells and these findings have sparked the search for glycan based biomarkers for the detection of different types of cancer [6]–[9]. In human hepatocarcinoma cells, the alterations of N-glycan structure in surface of glycoproteins contribute to the alterations in metastasis-associated phenotypes [10], [11]. Sakuma et al reported that an α1, 6-fucosylated biantennary N-glycan structure correlates with pulmonary metastatic ability of cancer cells [12]. In the work of Granovsky *et al*, the importance of specific glycosylation events in mammary cancer metastases has been clearly demonstrated *in vivo* using genetically altered mice [13]. These findings suggest that glycosylation may be involved in the regulation of multiple aspects of tumor metastasis.

The murine hepatocarcinoma cell lines Hca-F with a high lymphatic metastasis rate over 80% and Hca-P with a low lymphatic metastasis rate less than 30% have been derived from 615-mice ascites-type hepatocarcinoma cell lines H_22_ [14]. Hca-F and Hca-P cells metastasize only to the lymph nodes, and not to other organs [15]. However, the relationship between glycosylation modification and lymphatic metastasis of murine hepatocarcinoma cells is still not clear.

In the current study, we compared the N-glycan composition profiling, expression of glycogenes and lectin binding profiling between Hca-F and Hca-P cell lines. Meanwhile, we mainly focused on the modification of N-glycan of cell surface to further address the important roles of glycosylation in lymphatic metastasis of murine hepatocarcinoma cells.

## Results

### MALDI-MS Analysis of N-glycan Composition Profiling from Hca-F and Hca-P Cells

MALDI-TOF MS analysis was utilized to evaluate the N-glycan composition profiling of Hca-F and Hca-P cell lines. Fig. 1 showed the MS spectra of N-glycans released from cell membranes and the observed MS signals of the N-glycans (peaks 1–34 in Fig. 1A) and the assigned N-glycan signals as were summarized in Table 1. The observed signal intensities in the mass spectra are presented as a histogram (Fig. 1B), with the estimated monosaccharide compositions. High mannoses analyzed in both cell lines were detected at peak 5, 7, 11, 15, and 17 (Table 1). Several major N-glycan differences of cell membrane derived from Hca-F and Hca-P were detected. Peak 10, 26 were detected exclusively in the Hca-F cell line. Peak 29 was detected exclusively in Hca-P cell line. Furthermore there were some differences regarding the intensities of all peaks in the spectra recorded from pools of Hca-F and Hca-P samples. Among those oligosaccharides, peak 1, 2, 3, 4, 5, 6, 7 and 34 increased in high lymphatic metastasis cell line Hca-F, and peak 25, 30 increased in low lymphatic metastasis cell line Hca-P. These data indicated that differential N-glycan composition might be associated with tumor lymphatic metastasis.

**Figure 1:** N-glycans composition profiling of Hca-F and Hca-P cell lines using Mass spectrometry analysis. (A) MALDI-TOF MS spectra of N-glycans released from membrane protein of Hca-F and Hca-P cell lines. (B) Histograms of relative intensities of the N-glycan signals observed. Values are the mean ± S.D of three permethylated samples from N-glycan samples. The signal numbers correspond to those described in Table 1.

**Table 1:** Summary of N-glycan in N-glycan in Hca-F and Hca-P cell lines identified by MALDI-TOF MS.

Peak no.	Observed *m/z*		Composition					
	Hca-F	Hca-P	Hex	HexNAc	Man	GlcNAc	NeuAc	Deoxyhexose
1	1171.69	1171.84	0	0	3	2	0	0
2	1345.85	1345.86	0	0	3	2	0	1
3	1375.89	1375.87	1	0	3	2	0	0
4	1416.89	1416.91	0	1	3	2	0	0
5	1579.94	1579.97	0	0	5	2	0	0
6	1591.01	1591.03	0	1	3	2	0	1
7	1784.07	1784.10	0	0	6	2	0	0
8	1795.18	1795.10	1	1	3	2	0	1
9	1836.12	1836.20	0	2	3	2	0	1
10	1982.22	No	1	1	3	2	1	0
11	1988.15	1988.20	0	0	7	2	0	0
12	1999.17	1999.28	2	1	3	2	0	1
13	2156.28	2156.27	1	1	3	2	1	1
14	2186.29	2186.30	2	1	3	2	1	0
15	2192.26	2192.30	0	0	8	2	0	0
16	2244.28	2244.34	2	2	3	2	0	1
17	2396.29	2396.37	0	0	9	2	0	0
18	2431.29	2431.41	2	2	3	2	1	0
19	2448.31	2448.42	3	2	3	2	0	1
20	2478.54	2478.44	4	2	3	2	0	0
21	2605.39	2605.47	2	2	3	2	1	1
22	2635.37	2635.44	3	2	3	2	1	0
23	2652.39	2652.50	4	2	3	2	0	1
24	2779.33	2779.57	2	2	3	2	1	2
25	2809.42	2809.56	3	2	3	2	1	1
26	2817.27	No	0	6	3	2	0	1
27	2839.35	2839.57	4	2	3	2	1	0
28	2897.47	2897.60	4	3	3	2	0	1
29	No	2938.68	3	4	3	2	0	1
30	2966.47	2966.65	2	2	3	2	2	1
31	2996.56	2996.64	3	2	3	2	2	0
32	3102.34	3101.89	5	3	3	2	0	1
33	3305.43	3305.77	6	3	3	2	0	1
34	3463.61	3463.19	5	3	3	2	1	1

The N-glycan were observed as [M+Na]+.

Hex, hexose; HexNAc, N-acetylhexosamine; Man, mannose; GlcNAc, N-actylglucosamine; NeuAc, N-acetylneuraminic acid.

### Differential Expression of Glycogenes in Hca-F and Hca-P Cell Lines

To evaluate the expression profile of glycogenes in high (Hca-F) and low (Hca-P) metastatic potential cells, a real-time RT-PCR analysis was performed. 9 genes (out of 62) were differentially expressed between the two cell lines. Six glycogenes, ST6GAL1, MGAT5, FUT8, B4GALT1, B3GALT1, and B3GNT8 were expressed at a higher level in Hca-F compared with those in Hca-P cells (i.e., >3-fold higher, Fig. 2A). Conversely, three glycogenes, CHST13, MGAT3, and ST8SIA were expressed at an elevated level (i.e., >3-fold higher, Fig. 2A) in Hca-P compared with the ones in Hca-F cells. Western blot analysis further confirmed the enzyme expression on Hca-F and Hca-P cells at protein level (Fig. 2B). These data indicated that differential glycogene expressions might be associated with lymphatic metastasis of murine hepatocarcinoma cells.

**Figure 2:** Differential expression of glycogenes in Hca-F and Hca-P cell lines. (A) The mRNA levels of glycogenes analyzed by real-time RT-PCR. The relative amount of glycogenes mRNA levels was normalized to GAPDH levels. Relative intensities ratio (>3-fold) of the glycogenes signals were observed. (B) Western blot analysis for enzyme was assessed. Data are the means ± SD of triplicate determinants.

### Differential FITC–lectin Binding Profiles of Hca-F and Hca-P Cell Lines with Flow Cytometry

To investigate the glycan profiles of cell surface from Hca-F and Hca-P cell lines, flow cytometry analysis was used observing fluorescence intensity. Fig. 3 shows that the obvious differences in fluorescence intensity for glycosylation were evident by comparison between the Hca-F and Hca-P cell lines as summarized below: (1) higher signals of SNA (Siaα 2-6Gal/GalNAc) in Hca-F cells, (2) higher fucosylation at the innermost GlcNAc in Hca-F cells as revealed by fluorescence intensity on LCA, (3) increased level of branching of N-glycans in Hca-F cells estimated by fluorescence intensity of L-PHA (Tri- and tetra-antennary complex oligosaccharides), ABA (Galβ1-3GalNAcα-Thr/Ser (T) and sialyl-T), and DSA ((GlcNAc)_n_, polyLacNAc and LacNAc (NA3, NA4)), (4) higher signals of E-PHA (NA2 and bisecting GlcNAc) in Hca-P cells (Fig. 3A, 3B). These results correlated well with the real-time PCR analysis of glycogene expression. High expressions of glycogenes are corresponding with high fluorescence intensity of lectins in both cell lines (Fig. 3C).

**Figure 3:** Differential FITC–lectin binding profiles of Hca-F and Hca-P cell lines using flow cytometry. (A) Histograms of fluorescence intensities of cells with specific carbohydrate expression as determined by flow cytometry using 7 different lectins. (B) The data are means ± SD of 3 independent assays of Hca-F and Hca-P cell lines, *P<0.05. (C) List of glycogenes responsible for lectin signals in Hca-F and Hca-P cell lines.

### N-glycosylation Modification Mediates the Invasive Ability of Hca-F Cells both in vitro and in vivo

To test directly whether the N-glycosylation of Hca-F cells influenced cells invasive ability, the modification of N-glycosylation was finished. Tunicamycin (TM), an inhibitor of endogenous N-glycosylation of newly synthesized proteins, has effect on N-glycan of Hca-F cells. CD147 is a highly N-glycosylated immunoglobulin superfamily transmembrane protein that is composed of two extracellular Ig domains, which contributes to a highly N-glycosylated form, HG-CD147 (∼40–60 kDa) and lowly glycosylated form, LG-CD147 (∼32 kDa) [19]. Treatment of Hca-F cells, with TM at a dose dependent (0, 1, 5, and 10 mg/ml) for 12 h, showed that N-glycosylation was highly sensitive to inhibition by TM. The CD147 (40 kDa) completely disappeared, and the level of the CD147 (40–60 kDa) was decreased. The 27 kDa band that appeared was consistent with the size of the core protein. The fraction of CD147 remaining at 60 kDa was likely synthesized before TM treatment. In addition, aliquots of membrane fractions of Hca-F cells were also exposed to exogenous PNGase F (Fig. 4A) to achieve deglycosylation. The CD147 (40–60 kDa) completely disappeared, and a 27–33 kDa band appeared. These results suggested that the N-glycosylation process in Hca-F cells was highly sensitive to inhibition by TM and PNGase F.

**Figure 4:** N-glycosylation modification mediates the invasive ability of Hca-F cells both in vitro and in vivo. (A) Western blot analysis of CD147 was performed using total membrane protein extracts. Hca-F cells were exposed to TM or PNGase F and then harvested for western blot analysis. Controls are Na^+^/K^+^-ATPase. Hca-F cells were treated with TM (B) or PNGase F (C) and thereafter the cell invasive ability was assessed by ECMatrix gel analysis in vitro. Hca-F cells were treated with TM (D, fluorescence; ×100) or PNGase F (F, fluorescence; ×100) and thereafter the cell invasive ability to peripheral lymph nodes was analyzed in vivo. The number of TM pre-treated (E) or PNGase F pre-treated (G) CFSE^+^Hca-F cells invasion to peripheral lymph nodes was measured by flow cytometry. Surface labeling was expressed as the percentage of positive cells in CFSE^+^Hca-F cells relative to the total number of analyzed cells (*P<0.05). The data were obtained from three independent experiments.

To examine whether the modification of N-glycosylation in Hca-F cells affected the invasive ability, we performed an in vitro ECMatrix gel analysis. Under TM and PNGase F treatment, the Hca-F cells showed decreased invasive ability, as compared with the Hca-F groups in the absence of TM and PNGase F (Fig. 4B, 4C).

The influence of glycosylation modification on the invasive ability of Hca-F cells to peripheral lymph nodes in vivo was determined in order to explore the potential involvement of glycosylation during tumor cells invasion. Under TM and PNGase F treatment, the Hca-F cells were labeled with CFSE. The invasive ability of CFSE-tagged cells in TM or PNGase F-treated groups to lymph nodes was reduced obviously, as compared with the Hca-F groups in the absence of TM and PNGase F in vivo (Fig. 4D, 4F).

To further investigate the positive ratio of CFSE-tagged cells in whole lymph node digest mixture, a flow cytometry analysis was carried out. As shown in Fig. 4E, 4G, the number of CFSE-tagged Hca-F cells in control, TM or PNGase F-treated groups were quite different. The Hca-F in the absence of TM and PNGase F -treated positive cells were 17.55% and 17.28%, but TM (10 µg/ml) and PNGase F-treated (24 hour) positive cells were only 10.81% and 9.57%. These observations supported that the modification of N-glycosylation could be associated with the invasive ability of murine hepatocarcinoma cells.

### Silence of ST6GAL1 Effects on the Invasive Ability of Hca-F Cells both in vitro and in vivo

ST6GAL1 glycogene encodes the β-galactoside α-2, 6-sialyltransferase 1, which catalyzes the transfer of sialic acid residue in α-2, 6-linkage to terminal galactose of glycan chains. Fig. 2A has showed that glycogene ST6GAL1 was expressed at a higher level (4.66-fold) in Hca-F compared with those in Hca-P cells. We silenced, by siRNA, in order to elucidate the direct implication glycogene in the lymphatic metastasis-related phenotypes of Hca-F cells. As shown in Fig. 5A, ST6GAL1 expression at protein level was down-regulated in ST6GAL1 transfectants compared with Hca-F-control siRNA transfectants. The cell invasion was determined using the Transwell assay. Interestingly, knockdown of ST6GAL1 expression significantly inhibited Hca-F-ST6GAL1 siRNA cells invasion relative to the Hca-F-control siRNA cells (Fig. 5B).

**Figure 5:** Silence of ST6GAL1 effects on the invasive ability of Hca-F cells both in vitro and in vivo. (A) Silencing of ST6GAL1 in Hca-F cells was analyzed by RNAi approach. After Hca-F cells were transfected with ST6GAL1 siRNA for 30 h, western blot analysis for ST6GAL1 was assessed. GAPDH was also examined and served as controls for sample loading. Relative signal intensities of ST6GAL1 protein levels were normalized against those of GAPDH by LabWorks (TM ver4.6, UVP, BioImaging systems) analysis, respectively (*P<0.05). (B) In vitro ECMatrix gel analysis is performed. The average number of cells that invaded through the filter was counted. Hca-F-ST6GAL1 siRNA cells were significantly less invasive (*P<0.05) than the Hca-F and Hca-F-control siRNA cells. (C, fluorescence; ×100) The results of ST6GAL1 siRNA-transfected CFSE^+^Hca-F cells invasion to lymph nodes were analyzed. The number of Hca-F-ST6GAL1 siRNA cells was decreased, compared with the Hca-F-control siRNA, Hca-F cells after 24 h. (D) The number of ST6GAL1 siRNA-transfected CFSE^+^Hca-F cells invasion to lymph nodes was measured by flow cytometry. Surface labeling was expressed as the percentage of positive cells relative to the total number of analyzed cells (*P<0.05). (E) FITC-SNA binding profiles of Hca-F cells using flow cytometry. Histograms of fluorescence intensities of cells with specific carbohydrate expression as determined. Data are the average ± SD of triplicate determinants.

The influence of glycogene on the invasive ability of Hca-F cells to peripheral lymph nodes in vivo was determined. Hca-F cells were labeled with CFSE, a green fluorescence dye, which can be transported across plasma membrane to react covalently with free amino group of intracellular macromolecules. The invasive ability of CFSE-tagged cells in ST6GAL1 siRNA-treated groups to lymph nodes was reduced obviously, as compared with control groups in vivo (Fig. 5C). To further investigate the positive ratio of CFSE-tagged cells in whole lymph node digest mixture, a flow cytometry analysis was carried out. As shown in Fig. 5D, the number of CFSE-tagged Hca-F cells in control, siRNA-treated groups were quite different. The Hca-F, control siRNA-treated positive cells were 17.21% and 17.52%, but ST6GAL1 siRNA-treated positive cells were only 8.95%. These observations supported that ST6GAL1 on Hca-F cells could play an important role in invasion to peripheral lymph nodes in vivo, and might therefore contribute to tumor lymphatic metastasis.

In order to evaluate whether ST6GAL1 silencing could modify the N-glycosylation profile in terms of α-2, 6-linked sialic acid using a flow cytometry, each cell group was bind with SNA lectin. Fig. 5E showed that the ST6GAL1 knockdown resulted in a decrease of fluorescence intensity compared with the control cells.

### Overexpression of ST6GAL1 Influences the Invasive Ability of Hca-P Cells both in vitro and in vivo

To explore the effect of ST6GAL1 on invasive ability, an Hca-P cell line transient expressing ST6GAL1 was established. It was found that the level of ST6GAL1 protein was notably increased in Hca-P transfectants (Fig. 6A). Furthermore, over-expression of ST6GAL1 significantly promoted Hca-P/ST6GAL1 cells invasion relative to the Hca-P/mock cells in vitro (Fig. 6B).

**Figure 6:** Overexpression of ST6GAL1 influences the invasive ability of Hca-P cells both in vitro and in vivo. (A) Hca-P cells were transfected with a pcDNA3.1 expression vector, and western blot analysis for ST6GAL1 was assessed. GAPDH was also examined and served as controls for sample loading. Relative signal intensities of ST6GAL1 protein levels were normalized against those of GAPDH by LabWorks (TM ver4.6, UVP, BioImaging systems) analysis, respectively (*P<0.05). (B) In vitro ECMatrix gel analysis is performed. The average number of cells that invaded through the filter was counted. Hca-P/ST6GAL1 cells were significantly more invasive (*P<0.05) than the Hca-P and Hca-P/mock cells. (C, fluorescence; ×100) The results of ST6GAL1-transfected CFSE^+^Hca-P cells invasion to lymph nodes were analyzed. The number of Hca-P/ST6GAL1 cells was increased, compared with the Hca-P/mock, Hca-P cells after 24 h. (D) The number of ST6GAL1-transfected CFSE^+^Hca-P cells invasion to lymph nodes was measured by flow cytometry. Surface labeling was expressed as the percentage of positive cells relative to the total number of analyzed cells (*P<0.05). (E) FITC-SNA binding profiles of Hca-P cells using flow cytometry. Histograms of fluorescence intensities of cells with specific carbohydrate expression as determined. Data are the average ± SD of triplicate determinants.

The effect of glycogene ST6GAL1 on the invasive ability of Hca-P cells to peripheral lymph nodes in vivo was also analyzed. The invasive ability to peripheral lymph nodes in vivo of CFSE-tagged cells in Hca-P/ST6GAL1 groups to lymph nodes was increased obviously, as compared with Hca-P/mock groups in vivo (Fig. 6C). The flow cytometry analysis showed that the positive ratio of CFSE-tagged cells in whole lymph node digest mixture was different. Hca-P/ST6GAL1 positive cells showed increased ratio, as compared with the Hca-P/mock groups (Fig. 6D).

Fig. 6E showed that the ST6GAL1 over-expression resulted in an increase of fluorescence intensity compared with the Hca-P/mock cells. These results clearly showed that glycogene ST6GAL1 was associated with lymphatic metastasis of murine hepatocarcinoma cells, thus suggesting the involvement of the lymphatic metastasis in the altered glycosylation profiles.

## Discussion

In the present study, we investigated the possible correlation of glycosylation modification and the tumor lymphatic metastasis in murine hepatocarcinoma cell lines Hca-F and Hca-P with high, low metastatic potential to lymph nodes.

The structural scheme of glycans is dependent on their compositions. MALDI-MS technology as a novel methodology provides high sensitivity and more rapid glycan analysis [20], [21], [22]. Zhang et al indicated that MS technology could facilitate the discovery of a novel and quantitative prognostic biomarker for gastric cancer with lymph node involvement [23].Three glycans were shown to provide good sensitivity and specificity for the separation of serum samples from patients with hepatocellular carcinoma and controls by MS technology [24]. In the current study, we compared the total N-glycans from Hca-F and Hca-P cell lines, and found dramatic differences in N-glycan profiles between these two groups (Fig. 1, Table 1). Peak 2, 6, 26, 34 corresponded to fucosylated oligosaccharides, and peak 10, 34 corresponded to sialylated oligosaccharides originating from Hca-F cells showed a significant increase. Moreover, major peaks 25, 30 corresponded to fucosylated and sialylated oligosaccharides originating from Hca-P cells also showed a significant increase. Therefore, monitoring of the N-glycan profile would be an important step in the prevention of tumor metastasis and would increase our understanding of metastasis mechanisms.

Oligosaccharides on glycoproteins are altered in tumorigenesis, and they often play a role in the regulation of the biological characteristics of tumors [25], [26]. Each oligosaccharide is synthesized by a specific glycosyltransferase. Glycogenes, which encode glycosyltransferases, are involved in glycan synthesis and modification. The current study clearly showed that the glycogene expressions were highly regulated, with 9 (out of 62) glycogenes (at least 3-fold, Table 1) significantly differentially expressed among the two cell lines. For example, ST6GAL1, which is significantly expressed at an elevated level (4.66-fold higher) in Hca-F compared with Hca-P cells, encodes β-galactosamide: α-2, 6-sialyltranferase 1 that is a key enzyme in the formation of sialic acid residue in α-2, 6-linkage to terminal galactose of glycan chains [27]. The result was consistent with the MALDI-TOF MS analysis, and a higher level of sialylated oligosaccharides in Hca-F cells was displayed (Fig. 1 and Table1). Therefore, the major altering expressions of glycogenes in the two cell lines may be more important as indicators and functional contributors of tumor lymphatic metastasis.

Lectin binding approache has been used for the analysis of glycoproteins and N-glycans [28]. Previous report [29] revealed lectin binding profiles of SSEA-4 enriched, pluripotent human embryonic stem cell surfaces using flow cytometry assay. In this study, the obtained datasets could be statistically compared to identify lectins that show significant differences between the two cell lines (Fig. 3A, 3B). For example, SNA specifically recognized α-2, 6-linked sialic acid and a higher signal of SNA for N-glycosylation in Hca-F cells was shown. High expression of glycogene ST6GAL1 was responsible for high fluorescence intensity of SNA FITC-lectin (Fig, 3C). The result was consistent with the MALDI-TOF MS and glycogene expression analysis.

The alterations in glycosylation can be associated with tumor either as a product of the tumor or as reaction to the disease [30], [31]. Inhibition of N-glycan processing disrupts normal cell adhesion and reduces the tumourigenic and metastatic capacity in vivo of rhabdomyosarcoma cell line S4MH [32]. Deglycosylation of Hca-F cells by tunicamycin influences on cells adhesion in vitro [33]. The CD147 gene has garnered attention because of its high expression in many malignant tumor cells, and its key role is in the processes of tumor progression [34]. In this study, we modified the N-glycosylation of Hca-F cells by tunicamycin or PNGase F treatment. Both treatments resulted in similar effects on the occurrence of a defective N-glycosylation in Hca-F cells. The altered N-glycosylation of CD147 were found in Hca-F cells, and further suggested a link between defective N-glycosylation of Hca-F cells and tumor invasion both in vitro and in vivo (Fig. 4). The detection of such strongly correlated glycosylation modification showed that not only glycan structure might alter, but that often tumor biological processes were affected.

Increased expression of ST6GAL1 is reported in carcinomas of the colon, breast, ovarian and gastric cancer, acute myeloid leukemia, and in some brain tumors [35]–[40]. ST6GAL1 is also correlated with invasion in cancers [41], [42], [43]. Altered expression of ST6GAL1 mediates the adhesive capability of Hca-F cells to fibronectin [44]. Our data proved the glycogene ST6GAL1 as potential target for tumor lymphatic metastasis. In addition, we further tested directly that the silencing of ST6GAL1 in Hca-F cells resulted in decreased the invasive ability both *in vitro and in vivo* through modifying the N-glycosylation profile in terms of α-2, 6-linked sialic acid in murine hepatocarcinoma cells (Fig. 5). ST6GAL1 product also decreased remarkably in Hca-F- ST6GAL1 siRNA cells labeled with SNA lectin. Conversely, over expression of ST6GAL1 in Hca-P cells could increase the invasive ability both *in vitro and in vivo* (Fig. 6). These observations clearly demonstrate that the changes in glycogene expression levels have impact in the remodeling of cell surface glycosylation, which may consequently affect the biological functions of tumor cells such as tumor lymphatic metastasis.

In conclusion, by analyzing the glycomics of Hca-F and Hca-P lines and detecting the quantitative changes of glycosylation, at least in this system, altered glycosylation showed the unusual property of association with tumor lymphatic metastasis. Although we feel that the modification of glycosylation effects remain the best explanation for the phenotype, there could be other potential effects on multiple glycomic alterations. Therefore, the molecular bases of tumor lymphatic metastasis-associated phenotype remains to be further investigated.

## Materials and Methods

### Cells

Murine hepatocarcinoma cell lines Hca-F and Hca-P, which have high, low metastatic potential in the lymph nodes, (established and stored by Department of Pathology, Dalian Medical University, Dalian) were implanted in mouse abdominal cavity [16]. After 7 days, all mice were sacrificed and cells were retrieved from the abdominal cavity by 10 mL syringe. Then cells were cultured 1 day in 90% RPMI 1640 (Gibco) supplemented with antibiotics (1× penicillin/streptomycin 100 U/ml, Gibco), 10% fetal bovine serum (Gibco), at 37°C in a humidified atmosphere containing 5% CO2. This study was carried out in strict accordance with the recommendations in the Guide for the Care and Use of Laboratory Animals of the National Institutes of Health. The protocol was approved by the Committee on the Ethics of Animal Experiments of the Dalian Medical University, China (Permit Number: 12-569). All surgery was performed under sodium pentobarbital anesthesia, and all efforts were made to minimize suffering.

### Membrane Protein Extract

A total of 1×10^7^ cells were washed with phosphate buffered saline (PBS) and lysed on a plate with lysis and separation buffer containing a protease inhibitor cocktail. Cell membrane proteins were extracted from the cell suspension using a CelLytic MEM Protein Extraction kit (Sigma, St Louis, MO, USA). The membrane protein concentration was measured with a Micro BCA Protein Assay kit (PIERCE, Rockford, IL) and used for further experiments as described below.

### Release of N-glycans from Cell Membrane Proteins

Three 100 µg aliquots of lyophilized samples (cell membrane proteins) were first digested with trypsin (10 µg) and chymotrypsin (10 µg) dissolved in 25 mM ammonium bicarbonate (25 µL) at 37°C for 18 h. The digest was left in a water bath (85°C, 5 min) and after cooling N-linked oligosaccharides were released from peptides by treatment with PNGaseF enzyme (2 µL; 6 U) at 37°C (18 h) followed by Pronase digestion (10 µg) at 37°C (8 h). During the incubation time, the reaction sample was mixed occasionally. The released N-glycans were purified using an Oasis HLB cartridge (60 mg/3 ml; Waters) and then were lyophilized.

### MS Analysis

The mass spectra were carried out in reflectron positive ion mode with MALDI-TOF MS ((Bruker Corp., Billerica, MA, USA). To increase sensitivity and provide more informative fragmentation, the released glycans were permethylated [17], [18] and further characterized by MALDI-TOF MS. For the type of MALDI analysis of the permethylated glycans, 2, 5-DHB was used as the matrix. Values are the mean ± S.D of three permethylated samples from N-glycan samples. All MS spectra were obtained from Na+ adduct ions.

### Analysis of Glycogenes

Total RNA were isolated from Hca-F and Hca-P cells using an RNeasy Mini Kit (QIAGEN) and cDNA was synthesized using QuantiTect Reverse Transcription Kit (QIAGEN) from 5 µg of total RNA according to the manufacturer’s instruction. Real-time PCR amplification and analysis were performed on 7500 fast Real-time PCR System (Applied Biosystems) for 40 cycles (15 seconds at 95°C, 15 seconds at 60°C and 30 seconds at 72°C). All reactions were performed with QuantiTect SYBR Green PCR Kit (QIAGEN) according to the manufacturer's instruction. The sequences of the upstream and downstream primers were as follows: 5′-TGCGTGTGGAAGAAAGGGAGC-3′ and 5′-CTCCTGGCTCTTCGGCATCTG-3′ for ST6Gal 1; 5′-CCCTGGAAGTTGTCCTCTCA-3′ and 5′-TCCTCTGCCAGTGCC TTAAT-3′ for MGAT5; 5′-GGATTGCAAATTCCTGCCATTC-3′ and 5′-AACGTTGT CCCGGGTGTCA-3′ for FUT8; 5′-GGCGTCACCCTCGTCTATTA-3′ and 5′-GCCC TGCAGTGTAGAGGAGA-3′ for B4GALT1; 5′-ACCGTGACATCGTGGAAGTGG- 3′ and 5′-GGATGGTGGGCAGCGTGTC-3′ for B3GALT1; 5′-CGGCGCTATGGTG ACCTACTG-3′ and 5′-TCAGCAGCAGCAGGTCCTTG-3′ for B3GNT8; 5′-TACGA CTCACTATAGGGGCGACTA-3′ and 5′-CCCTCACTAAAGGGAGTCCTAGGA-3′ for CHST13; 5′-GCGTGATGGTGTGCTGTTCC-3′ and 5′-ACAGGGACTTCCGC A TGTGG-3′ for MGAT3; 5′-CCTAGCACAGGTCTCCTCATG-3′ and 5′-GGAAAT GGCCAGAATCCATA-3′ for ST8SIA4; 5′-ATTGCCCTCAACGACCACTT-3′ and 5′ -AGGTCCACCACCCTGTTGCT-3′ for GAPDH. Expression levels of each glycogene were normalized using either the expression level of GAPDH mRNA and compared between Hca-F and Hca-P cell lines. Real-time RT-PCR analysis was performed in triplicate.

### Flow Cytometry Assay

Hca-F and Hca-P cell lines were washed thrice with fluorescence-activated cell sorting (FACS) buffer (PBS containing 20 g/L bovine serum), and then centrifuged at 1000 r/min for 5 min in a 1.0 mL eppendorf tube for collecting cells. The cells were blocked for 30 min 37°C in 5% powdered skim milk and then were washed between each step with FACS buffer. Cells were placed in sterile conical tubes in aliquots of 500,000 cells each and stained with one of the 7 FITC-lectins at a final concentration of 10 µg/ml for 40 min at 4°C in the dark. Residual unbound FITC–lectin was then discarded by repeat centrifugation of samples at 1000 r/min. After removal of supernatant, cells were resuspended in 0.2 ml PBS. The control, which was negative, cells and FITC–lectins were alone. Fluorescence and light scatters were analyzed in a BD Biosciences fluorescence-activated cell sorter (FACSCalibur) equipped with an argon laser tuned at 488 nm and a 635-nm diode, and Cell Quest software was used for acquisition. Ten thousand cells were analyzed for each sample. Three independent assays were carried out using both Hca-F and Hca-P cell lines.

### RNAi Assay

Hca-F cells were incubated in appropriate antibiotic-free medium with 10% fetal bovine serum (Gibco), transferred to a 6 well tissue culture and incubated at 37°C, in a CO_2_ incubator to obtain 60–80% confluens. The cell cultures were transfected with ST6GAL1 siRNA Transfection Reagent Complex, respectively (Santa Cruz Biotech, Inc, sc-42805), which was prepared according to the protocol. Scrambled siRNA was used as the negative control. Transfer cells were cultured and incubated at 37°C for 6 hours, followed by incubation with complete medium for additional 24 h. Then cells were harvested and experimented as described for western blot analysis, in vitro and in vivo invasion assay. The cell transfection efficiency was 79% and the survival rate was 86%, respectively.

### Transfection

To generate ST6GAL1-transfected mouse hepatocarcinoma cell line Hca-P the coding region of wild-type ST6GAL1 was subcloned into pcDNA3.1 expression vector (Invitrogen) to generate pcDNA3.1/ST6GAL1. The plasmid was mixed with Lipofectamine™ 2000 (Invitrogen) according to manufacturer’s instructions and added to Hca-P cells. The transient transfectants were selected and used as a population assigned Hca-P/ST6GAL1. The empty vector was used as a transfection control and resulting transfeatants were assigned Hca-P/Mock. The cell transfection efficiency was 72% and the survival rate was 86%.

### Tunicamycin Treatment

To inhibit N-linked glycosylation of newly synthesized proteins, Hca-F cells were washed once with PBS and cultivated for 12 h in fresh culture media (90% DMEM supplemented with antibiotics) in the absence or presence of TM (Sigma Aldrich, St. Louis, MO) in a dose-dependent manner (0, 1, 5, or 10 µg/ml). The cells were washed with PBS again and then were determined by western blot analysis and invasion assay. The cell survival rates were 89%, 90%, 87% and 85% by trypan blue dye exclusion assay, respectively.

### PNGase F Treatment

To remove N-glycans, membrane protein fractions (100 µg) from Hca-F cells were deglycosylated with 25 units of PNGase F (PNGase F from Elizabethkingia meningoseptica; Sigma Aldrich, St. Louis, MO) in lysis buffer. The probes were incubated for 8, 16, 24 hours at 37°C. Afterwards, reactions were stopped with sample buffer and the proteins were separated in a gel as described earlier. Besides, for the deglycosylation of membrane proteins, intact Hca-F cells were incubated with 25 units of PNGase for 24 hour, washed and subsequently treated as described for western blot analysis, in vitro and in vivo invasion assay. The cell survival rate was 88%, 89%, 85% and 87% by trypan blue dye exclusion assay, respectively.

### Western Blot Analysis

Whole cell proteins were electrophoresed under reducing conditions in 10% polyacrylamide gels. The separated proteins were transferred to a polyvinylidene difluoride membrane. After blocking with 5% skimmed milk in PBS containing 0.1% Tween 20 (PBST), the membrane was incubated with antibody (Santa Cruz Biotech or Abcam) and then with peroxidase-conjugated anti-rabbit IgG (1/10000 diluted; GE Healthcare UK Ltd., Little Chalf-ont, U.K.). A Na^+^/K^+^-ATPase α1 antibody (1/200 diluted; Santa Cruz Biotech) or GAPDH (1/200 diluted; Santa Cruz Biotech) was used as a control. All bands were detected using ECL Western blot kit (Amersham Biosciences, UK), according to the manufacturer’s instruction. The bands were analyzed with LabWorks (TM ver4.6, UVP, BioImaging systems).

### In vitro ECM Invasion Assay

Cells invasion in vitro was demonstrated using 24-well transwell units (Corning, NY, USA) with 8 µm pore size polycarbonate filter coated with ECMatrix gel (Chemicon) to form a continuous thin layer (Zhu et al., 2005). Cells (3×10^5^) were harvested in serum-free medium containing 0.1% BSA and added to the upper chamber. The lower chamber contained 500 µl RPMI 1640. Cells were incubated for 24 h at 37°C, 5% CO_2_ incubator. At the end of incubation, the cells on the upper surface of the filter were completely removed by wiping with a cotton swab. Then the filters were fixed in methanol and were stained with Wright-Giemsa. Cells that had invaded the Matrigel and reached the lower surface of the filter were counted under a light microscope at a magnification of 400×. Triplicate samples were acquired and the data were expressed as the average cell number of 5 fields.

### In vivo Invasion Assay

Cells (5×10^6^) were labeled with the vital dye carboxyfluorescein diacetate succinimidyl ester (CFSE, Sigma), respectively (Chen et al., 2005). Cells were incubated with 5 µM CFSE at 37°C for 10 min. Labeled cells were washed once and counted. After 1 day, the cells were harvested, and inoculated into the footpad of mice subcutaneously. After 12 h, lymph nodes were removed from mice. The frozen sections of lymph nodes were analyzed under fluorescence microscope with the Image-Pro Plus 4.5 software (Media Cybernetics, Silver Spring, MD, USA). The lymph nodes were incubated with 0.1% (w/v) collagenase IV (Sigma), in 90% RPMI 1640 (Gibco) 10% FBS (Gibco) for 30 min at 37°C. The ratio of green fluorescence positive Hca-F cells in whole lymph node digest mixture was detected by flow cytometry. Experiments were approved by the Committee on the Ethics of Animal Experiments of the Dalian Medical University, China (Permit Number: 12-569).

### Statistical Analysis

Each experiment was performed at least in triplicate, and the measurements were performed in three independent experiments. Data are expressed as means ± standard deviation (SD). Student’s t-test was used to compare the means of two groups. P<0.05 was considered statistically significant. All analyses were performed using SPSS 13.0 statistical packages (SPSS Inc., Chicago, IL).

## References

[1] DwekRA (1995) Glycobiology: “towards understanding the function of sugars”. Biochem Soc Trans 23: 1–25.775865510.1042/bst0230001

[2] TaniguchiN, EkuniA, KoJH, MiyoshiE, IkedaY, et al (2001) A glycomic approach to the identification and characterization of glycoprotein function in cells transfected with glycosyltransferase genes. Proteomics 1: 239–247.1168087010.1002/1615-9861(200102)1:2<239::AID-PROT239>3.0.CO;2-K

[3] SaxonE, BertozziCR (2001) Annu. Chemical and biological strategies for engineering cell surface glycosylation. Rev Cell Dev Biol 17: 1–23.10.1146/annurev.cellbio.17.1.111687482

[4] OhtsuboK, MarthJD (2006) Glycosylation in cellular mechanisms of health and disease. Cell 126: 855–867.1695956610.1016/j.cell.2006.08.019

[5] DennisJW, GranovskyM, WarrenCE (1999) Glycoprotein glycosylation and cancer progression. Biochim Biophys Acta 1473: 21–34.1058012710.1016/s0304-4165(99)00167-1

[6] BalogCI, StavenhagenK, FungWL, KoelemanCA, McDonnellLA, et al (2012) N-glycosylation of colorectal cancer tissues: a liquid chromatography and mass spectrometry-based investigation. Mol Cell Proteomics 11: 571–585.2257387110.1074/mcp.M111.011601PMC3434767

[7] Dube DH BertozziCR (2005) Glycans in cancer and inflammation-potential for therapeutics and diagnostics. Nat Rev Drug Discov 4: 477–488.1593125710.1038/nrd1751

[8] MehtaA, NortonP, LiangH, ComunaleMA, WangM, et al (2012) Increased Levels of Tetra-antennary N-Linked Glycan but Not Core Fucosylation Are Associated with Hepatocellular Carcinoma Tissue. Cancer Epidemiol Biomarkers Prev 21: 925–933.2249031810.1158/1055-9965.EPI-11-1183PMC3380809

[9] de LeozML, YoungLJ, AnHJ, KronewitterSR, KimJ, et al (2011) High-mannose glycans are elevated during breast cancer progression. Mol Cell Proteomics 10: M110.002717.10.1074/mcp.M110.002717PMC301345321097542

[10] GuoHB, ZhangY, ChenHL (2001) Relationship between metastasis-associated phenotypes and N-glycan structure of surface glycoproteins in human hepatocarcinoma cells. J Cancer Res Clin Oncol 127: 231–236.1131525710.1007/s004320000186PMC12164942

[11] GuoR, ChengL, ZhaoY, ZhangJ, LiuC, et al (2013) Glycogenes mediate the invasive properties and chemosensitivity of human hepatocarcinoma cells. Int J Biochem Cell Bio 45: 347–358.2310383610.1016/j.biocel.2012.10.006

[12] SakumaK, FujimotoI, HitoshiS, TanakaF, IkedaT, et al (2006) An N-glycan structure correlates with pulmonary metastatic ability of cancer cells. Biochem Biophys Res Commun 340: 829–835.1638007610.1016/j.bbrc.2005.12.072

[13] GranovskyM, FataJ, PawlingJ, MullerWJ, KhokhaR, et al (2000) Suppression of tumor growth and metastsis in Mgat5-deficient mice. Nat Med 6: 306–312.1070023310.1038/73163

[14] HouL, LiY, JiaYH, WangB, XinY, et al (2001) Molecular mechanism about lymphogenous metastasis of hepatocarcinoma cells in mice. World J Gastroenterol 7: 532–536.1181982310.3748/wjg.v7.i4.532PMC4688667

[15] LiHF, LingMY, XieY, XieH (1998) Establishment of a lymph node metastatic model of mouse hepatocellular carcinoma Hca-F cells in C3H/Hej mice. Oncol Res 10: 569–573.10367938

[16] JiaL, WangS, ZhouH, HuY, ZhangJ (2006) Caveolin-1 upregulates CD147 glycosylation and the invasive capability of murine hepatocarcinoma cell lines. Int J Biochem Cell Biol 38: 1584–1593.1670202010.1016/j.biocel.2006.03.019

[17] CostelloCE, Contado-MillerJM, CipolloJF (2007) A glycomics platform for the analysis of permethylated oligosaccharide alditols. J Am Soc Mass Spectrom 18: 1799–1812.1771923510.1016/j.jasms.2007.07.016PMC4383468

[18] ViseuxN, CostelloCE, DomonB (1999) Post-source decay mass spectrometry: optimized calibration procedure and structural characterization of permethylated oligosaccharides. J Mass Spectrom 34: 364–376.1022636310.1002/(SICI)1096-9888(199904)34:4<364::AID-JMS787>3.0.CO;2-P

[19] TangW, ChangSB, HemlerME (2004) Links between CD147 Function, Glycosylation, and Caveolin-1. Molecular Biology of the Cell 15: 4043–4050.1520134110.1091/mbc.E04-05-0402PMC515339

[20] DellA, MorrisHR (2001) Glycoprotein Structure Determination by Mass Spectrometry. Science 291: 2351–2356.1126931510.1126/science.1058890

[21] HarveyDJ (2005) Proteomic analysis of glycosylation: structural determination of N-and O-linked glycans by mass spectrometry. Expert Rev Proteomics 2: 87–101.1596685510.1586/14789450.2.1.87

[22] ZaiaJ (2004) Mass spectrometry of oligosaccharides. Mass Spectro Rev 3: 161–227.10.1002/mas.1007314966796

[23] Zhang MH, Xu XH, Wang Y, Ling QX, Bi YT, et al.. (2013) A Prognostic Biomarker for Gastric Cancer With Lymph Node Metastases. Anat Rec (Hoboken) Feb 4 doi: 10.1002/ar.22642.10.1002/ar.2264223382154

[24] GoldmanR, RessomHW, VargheseRS, GoldmanL, BascugG, et al (2009) Detection of Hepatocellular Carcinoma Using Glycomic Analysis. Clin. Cancer Res 15: 1808–1813.10.1158/1078-0432.CCR-07-5261PMC285019819223512

[25] DwekRA (1996) Glycobiology: toward understanding the function of sugars. Chem Rev 96: 683–720.1184877010.1021/cr940283b

[26] VarkiA (1993) Biological roles of oligosaccharides: all of the theories are correct. Glycobiology 3: 97–130.849024610.1093/glycob/3.2.97PMC7108619

[27] Harduin-Lepers A. Vallejo-RuizV, Krzewinski-RecchiMA, Samyn-PetitB, JulienS, et al (2001) The human sialyltransferase family. Biochimie 83: 727–737.1153020410.1016/s0300-9084(01)01301-3

[28] HirabayashiJ (2004) Lectin-based structural glycomics: glycoproteomics and glycan profiling. Glycoconj J 21: 35–40.1546739610.1023/B:GLYC.0000043745.18988.a1

[29] VenableA, MitalipovaM, LyonsI, JonesK, ShinS, et al (2005) Lectin binding profiles of SSEA-4 enriched, pluripotent human embryonic stem cell surfaces. BMC Dev Biol 21: 5–15.10.1186/1471-213X-5-15PMC118236116033656

[30] Ruhaak LR, Miyamoto S, Lebrilla CB (2013) Developments in the identification of glycan biomarkers for the detection of cancer. Mol Cell Proteomics Jan 30. [Epub ahead of print].10.1074/mcp.R112.026799PMC361733123365456

[31] KimEH, MisekDE (2011) Glycoproteomics-based identification of cancer biomarkers. Int J Proteomics 2011: 601937.2208469110.1155/2011/601937PMC3195811

[32] CalleY, PalomaresT, CastroB, del OlmoM, BilbaoP, et al (2000) Tunicamycin treatment reduces intracellular glutathione levels: effect on the metastatic potential of the rhabdomyosarcoma cell line S4MH. Chemotherapy 46: 408–428.1105390710.1159/000007322

[33] JiaL, ZhouH, WangS, CaoJ, WeiW, et al (2006) Deglycosylation of CD147 down-regulates Matrix Metalloproteinase-11 expression and the adhesive capability of murine hepatocarcinoma cell HcaF in vitro. IUBMB Life 58: 209–216.1675429910.1080/15216540600719580

[34] MuramatsuT, MiyauchiT (2003) Basigin (CD147): a multifunctional transmembrane protein involved in reproduction, neural function, inflammation and tumor invasion. Histol and Histopathol 18: 981–987.10.14670/HH-18.98112792908

[35] GessnerP, RiedlS, QuentmaierA, KemmnerW (1993) Enhanced activity of CMP-NeuAc:Galh 1–4GlcNAc:a 2,6-sialyltransferase in metastasizing human colorectal tumor tissue and serum of tumor patients. Cancer Lett 75: 143–149.831334910.1016/0304-3835(93)90056-f

[36] RecchiMA, Harduin-LepersA, Boilly-MarerY, VerbertA, DelannoyP (1998) Multiplex RT-PCR method for the analysis of the expression of human sialyltransferases: application to breast cancer cells. 5: 19–27.10.1023/a:10069832149189530953

[37] LiJ, WangY, XieY, XuZ, YangJ, et al (2012) Altered mRNA expressions of sialyltransferases in human gastric cancer tissues. Med Oncol 29: 84–90.2114024210.1007/s12032-010-9771-1

[38] WangPH, LeeWL, JuangCM, YangYH, LoWH, et al (2005) Altered mRNA expressions of sialyltransferases in ovarian cancers. Gynecologic Oncology 99: 631–639.1611217810.1016/j.ygyno.2005.07.016

[39] SkacelPO, EdwardsAJ, HarrisonCT, WatkinsWM (1991) Enzymic control of the expression of the X determinant (CD15) in human myeloid cells during maturation: the regulatory role of 6′-sialyltransferase. Blood 78: 1452–1460.1679356

[40] KanekoY, YamamotoH, KerseyDS, ColleyKJ, LeestmaJE, et al (1996) The expression of Galh1,4GlcNAc a2,6 sialyltransferase and a2,6-linked sialoglycoconjugates in human brain tumors. Acta Neuropathol (Berl) 91: 284–292.883454110.1007/s004010050427

[41] LinS, KemmnerW, GrigullS, SchlagPM (2002) Cell surface alpha 2,6 sialylation affects adhesion of breast carcinoma cells. Exp Cell Res. 276: 101–110.10.1006/excr.2002.552111978012

[42] ChristieDR, ShaikhFM, LucasJA, BellisSL (2008) ST6Gal-I expression in ovarian cancer cells promotes an invasive phenotype by altering integrin glycosylation and function. J Ovarian Res 1: 3.1901465110.1186/1757-2215-1-3PMC2584051

[43] ZhuY, SrivatanaU, UllahA, GagnejaH, BerensonCS, et al (2001) Suppression of a sialyltransferase by antisense DNA reduces invasiveness of human colon cancer cells in vitro. Biochim Biophys Acta 1536: 148–160.1140635010.1016/s0925-4439(01)00044-8

[44] YuS, ZhangL, LiN, FanJ, LiuL, et al (2012) Caveolin-1 up-regulates ST6Gal-I to promote the adhesive capability of mouse hepatocarcinoma cells to fibronectin via FAK-mediated adhesion signaling. Biochem Biophys Res Commun 427: 506–512.2302219010.1016/j.bbrc.2012.09.086

